# Nanoemulsion and Encapsulation Strategy of Hydrophobic Oregano Essential Oil Increased Human Prostate Cancer Cell Death via Apoptosis by Attenuating Lipid Metabolism

This article has been retracted.

**DOI:** 10.1155/2022/9569226

**Published:** 2022-05-26

**Authors:** Haribalan Perumalsamy, Rajeshkumar Shanmugam, Jun-Ran Kim, Gokulanathan Anandapadmanaban, Md. Amdadul Huq, Kamal Dua, Dinesh Kumar Chellappan, Tae Hyun Yoon, Sri Renukadevi Balusamy

**Affiliations:** ^1^Institute for Next Generation Material Design, Hanyang University, Seoul 04763, Republic of Korea; ^2^Center for Creative Convergence Education, Hanyang University, Seoul 04763, Republic of Korea; ^3^Research Institute for Convergence of Basic Science, Hanyang University, Seoul 04763, Republic of Korea; ^4^Department of Pharmacology, Saveetha Dental College & Hospitals, Saveetha Institute of Medical and Technical Sciences (SIMATS), Chennai, Tamilnadu, India; ^5^Experiment & Analysis Division, Animal and Plant Quarantine Agency, Honam Regional Office, Jeollabuk-Do 540-96, Republic of Korea; ^6^Department of Food and Nutrition, Chung Ang University, Anseong-Si, Gyeonggi-Do 17546, Republic of Korea; ^7^Discipline of Pharmacy, Graduate School of Health, University of Technology, Sydney, Ultimo, NSW 2007, Australia; ^8^Faculty of Health, Australian Research Centre in Complementary and Integrative Medicine, University of Technology Sydney, Ultimo, NSW 2007, Australia; ^9^Uttaranchal Institute of Pharmaceutical Sciences, Uttaranchal University, Dehradun 248007, Uttarakhand, India; ^10^Department of Life Sciences, School of Pharmacy, International Medical University, Kuala Lumpur 57000, Malaysia; ^11^Department of Chemistry, College of Natural Sciences, Hanyang University, Seoul 04763, Republic of Korea; ^12^Department of Medical and Digital Engineering, College of Engineering, Hanyang University, Seoul, Republic of Korea; ^13^Department of Food Science and Biotechnology, Sejong University, Gwangjin-Gu, Seoul 05006, Republic of Korea

## Abstract

*Origanum vulgare* essential oil (EO) is traditionally well-known for its aromatic properties and biomedical applications, including anticancer. This was the first report where oregano essential oil-based nano emulsion (OENE) was synthesized for studying its effects on prostate cancer cell lines (PC3). At first, we have synthesized OENE and characterized using various spectroscopic analyses. The toxicity and inhibitory concentration (IC_50_) of OENE toward prostate cancer by MTT analysis were performed. The lipid biogenesis mediated, molecular target pathway analyses were performed using fluorescence cellular staining techniques, real-time RT-PCR, or western blotting analysis. OENE showed IC_50_ at 13.82 *µ*g/mL and significantly induced distinct morphological changes, including cell shrinkage, cell density, and cell shape reduction. In addition, OENE could also significantly decreased lipid droplet accumulation which was confirmed by studying mRNA transcripts of 3-hydroxy-3-methylglutaryl-CoA reductase (HMGCR) (0.31-fold), fatty acid synthase (FASN) (0.18-fold), and sterol regulatory element-binding protein (SREPB1) (0.11-fold), respectively. Furthermore, there is a significant upregulation BAX (BCL2 associated X) and caspase 3 expressions. Nevertheless, OENE decreased the transcript level of BCL2 (B-cell lymphoma 2), thus resulting in apoptosis. Overall, our present work demonstrated that OENE could be a therapeutic target for the treatment of prostate cancer and warrants in vivo studies.

## 1. Introduction

*Origanum vulgare* belongs to the family “Lamiaceae,” commonly known as oregano. The aromatic odor and flavor of the plant are due to the essential oil content. The spice of oregano is popularly used in the Mediterranean diet to treat and cure various health ailments, including anticancer [1–6]. The different species of Origanum showed cytotoxicity towards various cancer cell lines. For instance, the ethanol and ethyl acetate extract of *O. vulgare* showed a promising cytotoxic effect against breast cancer cell lines. Similarly, ethanolic extract of *O. compactum* also showed an antiproliferative effect on breast cancer cells. In addition, the ant-cancer effect was also reported on A549 (lung) and SMMC-7721 (hepatoma) cells, respectively [7, 8]. The inhibition of fatty acid biosynthesis and inducing apoptosis of cancer cell are crucial for the inhibition of cancer cell growth.

The metastatic feature of prostate cancer denotes the high-level expression of fatty acid (FA) and lipids biosynthesis [9–11]. The overexpression of FAS (Fas cell surface death receptor) derived from tumor tissue and cell lines denotes a well-grown metastatic stage of cancerous growth [12, 13]. Consequently, downregulation of fatty acid synthesis and induction of apoptosis using pharmacologically active biocompounds is crucial to inhibit cancer cell growth [14, 15]. The FAS expression is always downregulated in normal cells depending upon their cellular metabolism, and the downregulation of FAS in cells would lead to apoptotic cell death [16–18]. However, in cancer cells, the fatty acid biosynthesis is crucial as they need to sustain cell membrane biosynthesis during rapid proliferation, provides energy during metabolic stress conditions [19], and inhibit apoptosis. The fatty acid biosynthesis is regulated by various genes involved in the lipid biogenesis pathway, such as 3-hydroxy-3-methylglutaryl-CoA reductase (HMGCR), fatty acid synthase (FASN), and sterol regulatory element-binding protein 1 (SREPB1). For the induction of apoptosis, the suppression of SREPB1 expression in cancer cells would avoid proliferation [20]. The intrinsic apoptotic mediated pathway mechanism mainly involves BAX and BCL-2 apoptotic proteins. The release of cytochrome C in the cytoplasm from the mitochondrial outer membrane induces caspase proteins (caspase 9 and caspase 3) and promotes apoptotic mediated cell death.

Nanoemulsion is a type of transparent or semitransparent colloidal dispersion system whose particle size ranges from 10 to 100 nm. Encapsulation of essential oil (EO) with nanoemulsion improved long-term stability and bioavailability [21, 22] and thus can show improved biomedical applications. Recently, several OENE have been reported to show various applications in food and biomedical industries as antimicrobial agents, to treat cutaneous, lung and diseases [23]. However, very little is known about the anticancer effect of OENE. Therefore, our present study was designed to examine OENE role in lipid biosynthesis metabolism that promote apoptotic induction in PC3 cells. Our study concludes that OENE could be a strong therapeutic candidate to induce apoptosis in prostate cancer cells.

## 2. Materials and Methods

### 2.1. Reagents and Chemicals

The materials and cell culture medium used in this study were high standard and purchased commercially, as mentioned previously [24]. The surfactants used for this study and purchased are as follows: PEG-60 hydroxylated castor oil (Cremophor RH 40, BASF, Ludwigshafen, Germany) and polyoxyethylene 4-lauryl ether (Brij 30, Sigma-Aldrich, St Louis, MO, EUA).

### 2.2. Preparation of Nanoemulsions

The emulsion is prepared with a slight modification of as previously reported [25, 26], by mixing of 9.5% (W/W) of surfactant Cremophor RH40, 2.90% (W/W) of Brij30 with 6% (W/W) of oregano oil, and 4% (W/W) of sunflower oil with an appropriate amount of distilled water. The mixture of the pre-emulsified solution was placed with a magnetic stirrer at 4500 rpm, and the mixture was placed at a hot plate to 75°C for 2 min. Then, it was repeated with a magnetic stirrer at 10000 rpm and heated to 60°C for 8 minutes. Then, the mixture was stored at 25°C for 8 hours. Later, the ice-cooled emulsion was ultrasonicated with a 15-mm Dia prob horn tip with an amplitude of 65 microns in bench-scale probe sonicator at 25°C for 300 seconds with 10 seconds interval [27]. After homogenization, the emulsion was placed for storage for further cell cytotoxicity assays.

### 2.3. Physiological Characterization of Nanoemulsions

The synthesized nanoemulsions with no phase separation, demonstrating long-term stability, were taken for further analysis as described [28]. The prepared oregano nanoemulsions (OENE) were diluted in water to observe the characteristic peaks using UV-visible spectrophotometer Jasco V-630 (Jasco, Japan) with a 10-mm path length cuvette. The interior part structure of nano emulsions was characterized by optical microscopy LEICA DM2500 (Leica, Germany). The nanoemulsion droplets were kept on the glass slide and monitored through the optical microscope to determine the shape and size of the particles. The dispersion, homogeneity, and nano emulsion size were observed by dynamic light scattering (DLS) (Zetasizer Nano^Ⓡ^ Model S90; Malvern Instruments, UK) to determine the polydispersity index (PDI) of nanoemulsions. All measurement calculations were performed in triplicates.

### 2.4. Morphological Observation of Nanoemulsion

The size and shape of the oregano nano emulsions were characterized using a MERLIN Model HR FE-SEM (Carl Zeiss, Germany) [29]. The nanoemulsions were diluted in the ratio of 1 : 1 in DW. The samples were dropped onto a carbon-coated platinum grid and observed using a MERLIN Model HR FE-SEM (Carl Zeiss) for further processing analysis.

### 2.5. Identification of Active Constituents from Nanoemulsions

A 7890A gas chromatograph (Agilent, Wilmington, DE), equipped with a split injector and a flame ionization detection system, was used to separate and detect the constituents of OENE. The major constituents from nanoemulsions were identified by gas chromatography-mass spectrum analysis (GC-MS) compared with oregano oil alone. The GC-MS conditions for analyzing the samples were used as previously described [30].

### 2.6. Cell Proliferation Assay

The antiproliferative activity of OENE against human prostate cancer (PC3) was evaluated using an MTT assay as our previous study [31, 32].

### 2.7. Light Microscopy

As previously mentioned, the cell culture for light microscopic cytotoxicity observation was used [31, 33]. The cells were treated with or without OENE (0, 6.2, 12.5, 25, 50, and 100 *µ*g/mL) for 2 days. Positive control Cisplatin was similarly prepared to that of OENE. We used DMSO as a negative control. After 48 h treatment, the cell phenotypic characteristic of with or without treatment of PC3 cells was observed through a microscope (Leica DMIL LED, Wetzlar, Germany).

### 2.8. Oil Staining

The assay was performed as previously described by Balusamy et al. [31, 33] to measure the lipid content of the cells with or without treatment.

### 2.9. Apoptotic Cell Death Detection

As per the previous study [31, 33], OENE induced apoptosis was characterized by Hoechst staining 33342 and propidium iodide staining analysis was performed. Approximately 2 × 10^4^/well of PC3 cells were cultured in a Petridish, and apoptosis was studied using Hoechst staining. The cells were treated with 25 and 50 *μ*g/mL OENE based on MTT analysis except for the control. The detection of apoptosis exhibited fluorescence in PC3 cells was measured by Leica DMLB fluorescence microscope (Wetzlar, Germany).

### 2.10. DNA Fragmentation

The dose-dependent OENE was used to analyze DNA fragment content in a PC3 cell line (2 × 10^5^/well) performed as previously mentioned [31, 33]. After 24 h of OENE treatment, the genomic DNA was carried out as per manufacturer instruction (Gene All Biotech, Korea). The concentration was an equivalent amount of DNA (150 ng) mixed with loading buffer and run onto 1% agarose gel electrophoresis.

### 2.11. Real-Time PCR Analysis

RNA was extracted from PC3 cells with or without OENE treatment using TriZol reagent. An RT PreMix kit (Bioneer, Daejeon, Republic of Korea) was used at 65°C for 5 minutes to synthesize cDNA from 1 *µ*g of total RNA. This cDNA was used to polymerize the target gene. After that, qRT-PCR was performed, and the relative mRNA expression levels were obtained through a real-time rotation analyzer. Specific primers were used with SYBR^Ⓡ^ Green SensiMix plus Master Mix to express the mRNA levels. The sequence of the characteristic primers was listed (Table 1). Next, 1 *µ*L of cDNA, 2 *µ*L of cyber green reagent, and 2 *µ*L of primer (F : R = 1 : 1) were added to the reaction solution. The thermal reaction was maintained for 36 cycles at 95°C for 10 seconds, 60°C for 10 seconds, and 72°C for 20 seconds.

### 2.12. Western Blotting Analysis

PC3 cells were cultured in 100 mm coated culture dishes at 5 × 10^5^ cells/well for 24 h and then exposed to OENE for 24 h. The cells were washed 3 times with PBS (pH 7.0). To obtain the proteins, cells were treated with RIPA buffer for 1 hour and then centrifuged at 12,000 rpm for 20 minutes at 4°C. Western blot analysis was conducted as previously described [32]. Antibodies like anti-*β* actin, anti-BAX, BCL2, and secondary antibodies were used as mentioned previously [26].

### 2.13. Data Analysis

The inhibition concentration of (IC_50_) OENE was calculated and interpreted with untreated cell lines using GraphPad Prism 5 software program (GraphPad Software, La Jolla, CA). All other experiments were performed with three replicates, and the data are calculated with mean (±SE) value. The significant values of data represent as ^*∗*^*p* < 0.05, ^∗∗^*p* < 0.01, and ^∗∗∗^*p* < 0.001, respectively.

## 3. Results

### 3.1. Physical and Chemical Characterization of OENE

The prepared oregano nanoemulsion (OENE) was used for the various spectroscopic characteristic analyses (Figure 1). The OENE absorbance's spectra was assessed by UV-visible spectroscopy in the wavelength ranges from 200 to 800 nm. A significant sharp peak was observed in the UV spectrophotometer at the wavelength ranging from 260 to 280 nm for OENE. In contrast, multiple peaks were observed in oregano oil alone at a similar wavelength (Figure 1(a)). Sunflower oil is used as a surfactant and as a negative control. No peak was observed at a similar wavelength for sunflower oil (Figure 1(a)). The droplet size of the OENE is measured without dilution, as dilution may modify the structure. Microscopic observation of the OENE sample through optical microscope indicated that homogenized spherical particles spread uniformly throughout the solutions Figure 1(b). It indicates a well-formed OENE sample. The polydispersity index of OENE showed very low values ranging from 0.26 ± 0.045, indicating a homogenous dispersed system of droplets in OENE samples (Figure 1(c)).

The morphology of OENE sample is shown in Figure 2(a). SEM analysis indicated that oil droplets are surrounded by the polymeric surfactant forming a spherical shape with agglomeration. Likewise, it showed a consistently spreading structure with homogenous dispersion. The elemental analysis mapping designated that OENE sample has only organic elements without any other redundant metals (Figure 2(b)). GC-MS analyzed the identification of active constitutes from oregano oil and OENE sample. The GC-MS spectrum of oregano and OENE samples were showed major constituents such as carvacrol, methyl 9-methyl-tetra decanoate, o-cymene, and linalool. It indicates no alternation or changes in main active constituents even after synthesizing OENE (Figure 3).

### 3.2. OENE Suppressed Cell Growth in Prostate Cancer Cells (PC3)

The growth inhibition of cancer cells was compared with normal cells by treating different concentrations of OENE and MTT assay. The cisplatin was used as a positive control. Our results showed that OENE could significantly inhibit prostate cancer cells in a dose-dependent manner (Figures 4(a)–4(d)). The inhibition of PC3 proliferation after the treatment with OENE at different concentrations showed in Figures 4(a)–4(d). The IC_50_ value of OENE against PC3 cells is 13.82 *µ*g/mL The positive control cisplatin was found to be 22.08 *µ*g/mL, whereas the normal cell line (MRC-5) showed very less effective towards OENE (Figure 4(c)).

### 3.3. Morphological Characteristics Affected by OENE Treatment

The PC3 cells changes were observed with different concentrations of OENE treatment (Figure 4(d)). The dose-dependent treatment of OENE revealed cellular modification in PC3 cell lines, as shown in Figure 4(d). The cellular death with significant damages in PC3 cell line was observed at a different dose of OENE compared with nontreatment control shown notable features such as distinguished cell membrane with undamaged cytoplasmic organelles and prominent nucleus.

### 3.4. OENE Altered Lipid Biosynthesis

Lipid biosynthesis is an important characteristic of cancer cell proliferation. Oil staining analysis was performed to evaluate the lipid biosynthesis of both samples (with and without OENE treatment). The OENE treatment in PC3 cells showed notable lipid contents changes compared with untreated cells (Figure 5A1-3). It is clearly denoted that OENE induced lipids' biosynthesis inhibition which is the cause of cancer cell proliferation (Figure S1). The OENE treatment at different concentrations showed cellular proliferation inhibition by inhibiting lipid contents (Figure 5A2-3). The major genes involved in lipid biosynthesis, such as *fatty acid synthase (FASN), HMG-CoA reductase (HMGCR) and regulator of cholesterol, and fatty acid metabolism (SREPB1)*, were studied with or without the treatment of OENE (Figures 5(b)–5(d)). The OENE downregulates the expression of *FASN* (0.71- and 0.18 folds), *HMGCR* (0.31- and 0.18-folds), and *SREBP1* (0.31 and 0.18 folds) at a different concentration such as 25 *µ*g/mL and 50 *µ*g/mL, respectively.

### 3.5. OENE Induced PC3 Cell Apoptosis

The apoptotic mediated cell death was detected by using Hoechst and propidium iodide (PI) staining analysis. The OENE treated PC3 cell line showed a damaged outer cell membrane with increased fluorescence staining of prominent nuclei denoting cellular death (Figure 6(a)2-3). However, untreated PC3 cells showed no cellular damage, and there is least fluorescence staining mark observed in the nucleus (Figure 6(a)1). Likewise, PI staining was performed to detect cellular death induction of OENE in PC3 cells (Figure 6(b)1–3). The untreated cells showed no to minimum fluorescence staining of nucleus indicating no cellular damage (Figure 6(b)1). The cells treated with OENE showed significant cellular damage with fluorescence-stained nucleus indicating apoptotic cell death (Figure 6(b)2-3).

### 3.6. OENE Caused DNA Fragmentation in Prostate Cancer

The integrity of DNA in both untreated and treated cells was observed (Figures 7(a)-7(b)) in PC3 cells. The degradation of DNA was observed in OENE treated samples compared with untreated control cells (Figure 7(a)). The band intensity was analyzed and measured by an image analyzer with Quantity One software (Figure 7(b)).

### 3.7. OENE Treatment Increased BAX and Caspase 3 Levels and Decreased BCL2 Expression

The proapoptotic (*BAX*) and antiapoptotic genes (*BCL2*) in the molecular apoptotic mediated pathway were analyzed with or without treatment of OENE (Figures 7(c)–7(e)). The enhanced *BAX* expression and decreased *BCL2* (2.5-fold) observed the intrinsic mediated apoptotic pathway analysis. Further, cytochrome C was released through the activation of *BAX* and *caspase 3* activation, thus resulting in the apoptotic mediated cell death in PC3 cells (Figures 7(c)–7(e)). The apoptotic proteins expression of *BAX*, *BCL2* and *caspase 3* were also observed by the treatment of OENE in PC3 cells (Figure 7(f)). These data also showed with similar effect of apoptotic genes observed by qRT-PCR analysis.

## 4. Discussion

Various pharmacological aspects of oregano EO were recorded (*Origanum vulgare*) including antimicrobial, anticancer, and other food preservative properties apart from its use as a Mediterranean spice in many regions [26]. Only a few studies have been reported antiproliferative effects of oregano essential oil against cancers [9, 34, 35]; nevertheless, none of them have studied molecular targeting signaling pathway using oregano extract nor by using synthesized oregano oil-based nanoemulsion (OENE) to elucidate anticancer properties. For the first time, we have synthesized the OENE to increase its stability, bioavailability, and thus to enhance the anticancer properties. The combination of oil, surfactant, and an aqueous phase colloidal dispersions are nanoemulsions and will influence the therapeutic payload of the drug, physicochemical properties, particle size, and stability [36]. It would be used to empower precise pointing and extensive circulation time [37]. The characterization of synthesized OENE establishes the quality and colloidal formation of the oil-surfactant combination dispersions. Further, the nanoemulsion's oil droplet is critical for determining the formulation's stability and additionally, a significant impact on drug loading and efficacy of lipophilic–hydrophilic encapsulation [38]. Microscopic techniques are essential such as optical microscopy and scanning electron microscopy (SEM) required to demonstrate the nanoemulsions structure [39]. Furthermore, GC-MS results showed the presence of active compounds of oregano essential oil as carvacrol, methyl myristate, alpha-cymene, and linalool respectively. The active compounds in the prepared OENE were as same as oregano EO; however, OENE loaded methyl myristate efficiently compared to other active compounds. We have explored the OENE ability to undergo intrinsic pathway mediated apoptosis by inhibiting the proliferation of cancer cells *in vitro*. With the outburst of cellular toxicity to normal cell lines, most synthesized drugs have recently failed to succeed in cancer treatment. Henceforth, development of natural-based novel drugs for cancer treatment is necessary to overcome the current situation. To develop a cancer therapeutic target with fewer side effects, we established nanoemulsions using oregano essential oil.

The upregulation of lipid contents in cancer cells helps to improve proliferation and energy source for metabolism, mainly from the de novo synthesis [40]. The lipid biosynthesis enzyme-related genes such as *HMGCR, FASN*, and *SREPB1* are mainly involved in cancer cell growth and differentiation through downregulating *FAS* expression [41]. The lipid metabolism is mainly involved in cancer proliferation and takes to the metastatic stage. In this study, we studied the downregulation of lipid metabolism and induction of apoptosis on PC3 cells by changes in responsible genes, such as *HMGCR*, *FASN*, and *SREPB1* (Figure 3). Lipid biosynthesis are essential to promote the cell growth, maintain the cell membrane integrity, cell structure etc., during rapid proliferation of cancer cells. OENE targets lipid metabolism biosynthesis that resulted in the inhibition of cancer cell growth proliferation. It indicated that OENE could mainly target lipid biosynthesis and lead to apoptotic cell death. Based on our findings, OENE downregulated lipid metabolism via inhibiting fatty acid biosynthetic gene's expression and decreased fatty acid content.

To monitor the activation of the apoptosis pathway at the molecular level by treating OENE, we have studied the expression BAX, BCL2, and caspase 3 with or without OENE treatment. Our data conclude that OENE targets apoptotic genes in PC3 cells by decreasing the expression of the antiapoptotic gene BCL-2 and overexpressing the proapoptotic genes BAX and caspase 3 through the intrinsic mediated apoptotic pathway (Figure 8). Similar studies on oregano was reported in stomach, colon, and melanoma cancers [24, 42, 43]. Additionally, DNA fragmentation and nuclear staining (Hoechst and PI staining) clearly denoted cellular death caused by OENE in PC3 cells by damaging the cell membrane and cytoplasmic cell organelles compared to the untreated cells. The shrinkage of cellular organelles and damaged cell wall showed distinct phenotypical features of apoptotic cell death [41, 44].

In conclusion, we observed that OENE persuaded intrinsic mediated apoptosis by inhibiting cell growth, and lipid biosynthesis directed cellular death in PC3 cells by causing damage cell size shape, condensed nuclei, etc. (Figure 8). This study proposed that OENE can be a promising candidate for its novel synthetic approaches of hydrophobic essential oils to act as an anticancer drug carrier in vitro. It will be thought-provoking to approach *in vivo* animal model to assess similar efficacy for future therapeutic purposes.

## Figures and Tables

**Figure 1:** Characterization of OENE. (a) UV characterization of synthesized OENE compared with oregano EO and blank; (b) optical microscopical observation of OENE; (c) polydispersity index of OENE indicates that homogenous dispersed system of droplets in OENE.

**Figure 2:** Scanning electron microscopic observation. (a) SEM observation of synthesized OENE; (b) elemental map analysis of OENE with SEM images.

**Figure 3:** Gas chromatographic-mass spectrum (GC-MS) analysis of OENE: The GC and GC-MS spectrum showed major constituents and their relative abundance in both oregano EO (a) and OENE (b).

**Figure 4:** Antiproliferative activity of prostate cancer cells (PC3) with or without OENE treatment. (a) The photographic picture was taken after performance MTT assay with or without OENE treatment; (b) antiproliferative activity of OENE with dose-dependent treatment and the antiproliferative activity was denoted (%); (c) IC_50_ value of OENE in PC3 cells compared to that of positive control cisplatin. The cellular toxicity effect of OENE was also compared with normal cell line MRC-5; (d) cell morphology observation of PC3 was perceived using a phase-contrast microscope. The images are representative of three independent replicates. Each graph denotes the mean ± SE of triplicate experiments (^∗∗∗^*p* < 0.001 using Student's *t*-test).

**Figure 5:** OENE inhibited fatty acid biosynthesis of PC3. (a) Oil Red O staining was used to identify the lipid droplets in PC3. (b) The mRNA expression analysis of *HMGCR, FASN, and SREPB1* transcripts involved in the lipogenesis pathway was quantified. The *β*-actin was used as an internal control. Each bar represents the mean ± standard error of triplicate samples from three independent experiments (*p*=0.05, using Student's *t*-test).

**Figure 6:** OENE induced apoptosis in PC3 cells. (a) Hoechst staining of PC3 cells with or without OENE treatment. (b) PI staining with or without OENE treatment. In control cells, the cell membrane remained intact and does not allow cells to stain with the dye. However, the damaged cells were stained and indicated apoptotic cells.

**Figure 7:** DNA fragmentation assay. (a) Genomic DNA was isolated from treated and control groups and loaded on 1% agarose gel electrophoresis containing ethidium bromide. (b) The band intensity was measured using an image analyzer with Quantity One software; (C–F) alteration in genes and protein expression of the apoptotic pathway. Upon OENE treatment, (c) BAX (proapoptotic protein), (d) downregulation of BCL2 (antiapoptotic protein), and (e) upregulation of caspase 3; (f) the protein targets of BAX, BCL2, and caspase 3 with or without treatment of OENE.

**Figure 8:** Schematic representation of OENE induced apoptosis in prostate cancer *in vitro*. OENE inhibited the expression of *fatty acid synthase (FASN), cholesterol biosynthesis genes (HMGCR)*, and *regulatory protein SREPB1*. This might have resulted in cell growth inhibition, proliferation, and induced apoptosis. The induction of apoptosis was confirmed by monitoring BAX, BCL2, and caspase 3 protein expression.

**Table 1:** Primers listed in the present study.

S. no.	Genes	Forward primer (5′-3′)	Reverse primer (5′-3′)
1.	*HMGCR*	CTTGTTCATGCTCACAGTCG	ACCAGCATAGGTTCACGTCTA
2.	*FASN*	AACGGCAACCTGGTAGTGAG	GTGTCCATGAAGCTCACCCA
3.	*SREBP1*	GATGCGGAGAAGCTGCCTAT	GCTGTGTTGCAGAAAGCGAA
4.	*BAX*	TTCTGACGGCAACTTCAACTG	GTTCTGATCAGTTCCGGCA
5.	*BCL2*	AGCACTCCCGCCACAAAGA	GAGGCAAGCATAAGACTGG
6.	*β-Actin*	CATCACTATCGGCAATGAGC	GACAGCACTGTGTTGGCATA

## Data Availability

The data that support the findings of this study are available on request from the corresponding author.

## Supplementary Materials

Supplementary Materials Figure S1: overview of the study.
